# BMP9 Inhibits Proliferation and Metastasis of HER2-Positive SK-BR-3 Breast Cancer Cells through ERK1/2 and PI3K/AKT Pathways

This article has been retracted.

**DOI:** 10.1371/journal.pone.0096816

**Published:** 2014-05-07

**Authors:** Wei Ren, Yuehong Liu, Shaoheng Wan, Chang Fei, Wei Wang, Yingying Chen, Zhihui Zhang, Ting Wang, Jinshu Wang, Lan Zhou, Yaguang Weng, Tongchuan He, Yan Zhang

**Affiliations:** 1 Department of General Surgery, The First Affiliated Hospital of Chongqing Medical University, Chongqing, China; 2 Key Laboratory of Diagnostic Medicine designated by the Ministry of Education, Chongqing Medical University, Chongqing, China; 3 Molecular Oncology Laboratory, Department of Surgery, The University of Chicago Medical Center, Chicago, Illinois, United States of America; Dartmouth, United States of America

## Abstract

Bone morphogenetic protein 9 (BMP9), a member of TGF-β superfamily, is reported to inhibit the growth and migration of prostate cancer, osteosarcoma and triple-negative MDA-MB-231 breast cancer cells. However, little is known about the effect of on the biological behaviors of HER2-positive SK-BR-3 breast cancer cells and the underlying mechanisms. This study aimed to investigate the effects of BMP9 on the proliferation and metastasis of SK-BR-3 cells with BMP9 over-expression or BMP9 down-regulated expression. Results indicated that exogenously expressed BMP9 inhibited the proliferation and metastasis of SK-BR-3 cells while decreased endogenous BMP9 expression in SK-BR-3 cells promoted the proliferation and migration of breast cancer cells *in vitro* and *in vivo*. In SK-BR-3 cells with BMP9 over-expression, the phosphorylation of HER2, ERK1/2 and AKT was markedly suppressed and the HER2 expression decreased at both mRNA and protein levels, while opposite results were observed in SK-BR-3 cells with BMP9 knock down. When the phosphorylation of ERK1/2 and PI3K/AKT was inhibited by PD98059 and LY294002, respectively, the decreased proliferation and invasion induced by BMP9 knock down were eliminated. These findings suggest that BMP9 can inhibit the proliferation and metastasis of SK-BR-3 cells via inactivating ERK1/2 and PI3K/AKT signaling pathways. Thus, BMP9 may serve as a useful agent in the treatment of HER-2 positive breast cancer.

## Introduction

Breast cancer is one of the most common malignancies and the second leading cause of cancer related deaths in women. Breast cancer is a heterogeneous disease and can be classified into luminal A (ER+ or PR+, HER2−), luminal B (ER+ or PR+, HER2+), HER2-positve (ER− and PR−, HER2+), and triple negative (ER− and PR−, HER2−) subtypes [1]. Luminal B classification was defined as the results of immunohistochemistry with ER-positive or PR-positive and HER2-positive. [1] Breast cancer with different molecular subtypes exhibits distinct susceptibility to anticancer therapies. Therefore, it is necessary to explore effective strategies for the treatment of breast cancer [2].

HER2 is aberrantly up-regulated in approximately 30% of breast cancer patients which is correlated with a poor clinical prognosis and chemo-resistance, making HER2 as an important therapeutic target [3]–[5]. The major signaling pathways activated by HER2 include the MAPK and PI3K/AKT pathways [5]–[7], both of which have been shown to be critical for the growth, migration and survival of HER2-positive breast cancer cells. Trastuzumab, which effectively inhibits the HER2 mediated MAPK and PI3K/AKT pathways, is the first target agent approved for the treatment of HER2 positive breast cancer [8]–[12]. However, many HER2-positive breast cancer patients do not respond to or eventually progress after trastuzumab therapy [1]. Thus, it is imperative to explore the mechanisms underlying the resistance of breast cancer and to develop novel strategies for the treatment of breast cancer.

Bone morphogenetic proteins (BMPs) belong to the transforming growth factor-β (TGF-β) superfamily and consist of at least 20 members in human [13]. BMPs are originally identified as osteoinductive cytokines that can promote bone and cartilage formation *in vivo*. Recently, they have shown to play a significant role in the regulation of tumor development, progression and bone metastasis [14]. BMP9, a new member of the BMP family, has been shown as a pleiotropic cytokine and is implicated in the bone morphogenesis, functional differentiation, glucose homeostasis, iron homeostasis, and angiogenesis [15]. Recently, accumulating evidence [16], [17] shows that BMP9 plays important roles in the regulation of various cellular processes, including cell proliferation, migration, differentiation and apoptosis. Studies have shown that exogenous BMP9 can significantly inhibit the growth, adhesion, invasion, as well as migration of triple negative MDA-MB-231 breast cancer cells *in vitro* and *in vivo* [13]. However, the functions of BMP9 in HER2-positive breast cancer have not been investigated.

In the present study, the effects of BMP9 on the proliferation and metastasis of HER2-positive SK-BR-3 breast cancer cells as well as the underlying molecular mechanisms were investigated in BMP9 over-expressing and BMP9 knock down cells. Our results showed that BMP9 suppressed the proliferation and metastasis of SK-BR-3 cells *in vitro* and inhibited the tumor growth *in vivo* through inactivating MAPK and PI3K/AKT signaling pathways.

## Materials and Methods

The ethics committee of the First Affiliated Hospital of Chongqing Medical University has approves this research.

### Cell Culture

Human SK-BR-3 breast cancer cells (ACTT, USA) were kindly provided by Dr. Tong-chuan He in the University of Chicago Medical Center, USA, and the MDA-MB-231 breast cancer cells were purchased from the Shanghai Institute for Biological Sciences, Chinese Academy of Science, China. SK-BR-3 cells and MDA-MB-231 cells were separately maintained in DMEM and L15 medium supplemented with 10% fetal calf serum (FCS; Gibco), 100 U/ml penicillin and 100 µg/ml streptomycin at 37°C in an environment with and without CO_2_.

### Cell Infection by Recombinant Adenovirus

Recombinant adenovirus expressing BMP9 (AdBMP9) and adenovirus expressing green fluorescent protein (AdGFP) were kindly provided by Dr. Tong-chuan He in the University of Chicago Medical Center. Recombinant adenovirus interfering BMP9 (AdsiBMP9) and negative control adenovirus (AdsiNC) were generated previously using the AdEasy system [18].

SK-BR-3 cells were seeded into 6-well plate and infected with AdBMP9, AdGFP, AdsiBMP9, AdsiNC adenoviruses, respectively. The medium was refreshed 12 h later. The fluorescence was detected 36 h later. The recombinant SK-BR-3/BMP9 cells, SK-BR-3/GFP cells, SK-BR-3/siBMP9 cells and SK-BR-3/siNC cells were used in following experiments.

### Antibodies and Reagents

Antibodies against ERK1/2, phosphor-ERK1/2, p38, phosphor-p38, JNK, phosphor-JNK, AKT and phosphor-AKT were purchased from Cell Signaling Technology. Antibodies against HER2 and phosphor-HER2 were from ImmunoWay Biotechnology. Antibodies against BMP9 and β-actin, and inhibitors of ERK1/2 (PD98059) and PI3K/AKT (LY294002) were from Santa Cruz Biotechnology (USA).

### RNA Isolation and RT-PCR

Total RNA extraction was performed using the Trizol reagent (Invitrogen, Carlsbad, CA, USA). cDNA was amplified with 1 µg of total RNA using a Primer Script Kit (TaKaRa, Dalian, China). Primers used for RT-PCR of BMP9 and HER2 are shown in Table 1. The mRNA expression of target genes was normalized to those of GAPDH.

**Table 1:** Primers used for RT-PCR.

Gene	Primer sequence (5′-3′)	Product size (bp)
BMP9	Forward: CTGCCCTTCTTTGTTGTCTT	322
	Reverse: CCTTACACTCGTAGGCTTCATA	
HER2	Forward: ACACTGATAGACACCAACCGCTC	379
	Reverse: CGTCCGTAGAAAGGTAGTTGTAGG	
GAPDH	Forward: CAGCGACACCCACTCCTC	120
	Reverse: TGAGGTCCACCACCCTGT	

### Western Blot Assay

Different recombinant cells were collected and lysed with radio immunoprecipitation assay (RIPA) buffer. The lysate was centrifuged and the supernatant was denatured by boiling. The western blotting assay was performed as usual. The target proteins were detected using the Super Signal West Pico Chemiluminescent Substrate kit. Data were recorded and analyzed using the Bio-Rad Electrophoresis Documentation (Gel Doc 1000) and Quantity One version 4.5.0 (Bio-Rad, Hercules, CA, USA).

### Cell Proliferation Assay

Cell proliferation was analyzed by MTT assay as described previously [13]. The absorbance was measured daily for 5 days at 492 nm using a microplate reader. Each experiment was done in quintuplicate, and repeated three times. Then, a growth curve was delineated.

### Colony Formation Assay

Different recombinant cells were collected, seeded at 200 cells/well into a 6-well plate with and maintained in DMEM medium containing 10% FCS for 2 weeks. When colonies were observed, cells were washed twice with PBS and stained with Wright method. The colony forming rate was estimated as follow: (colony number/cell number)×100%. The experiment was repeated three times.

### Wound-closure Assay

SK-BR-3 cells (5×10^5^/well) were seeded into 6-well plate and maintained in DMEM containing 10% FCS for 8 h followed by treatment with different adenoviruses for 6 h. The medium was refreshed with DMEM containing 1% FCS. When the cell confluence reached 100%, a wound was created at the center with a sterile micropipette tip. Cell migration was monitored by microscopy 18 h later and reported as the estimated ratio of the remaining wounded area to the initial wound area. The experiment was done in triplicate.

### Transwell Invasion Assay

The invasion assay was performed as previously described (14). The chamber of a non-type I -coated 24-well culture insert (Millipore, Billerica, MA, USA) was used, and the upper chamber of the insert was coated with extracellular matrix (ECM) gel (Sigma, St. Louis, MO, USA). The recombinant cells infected with different adenoviruses were seeded into the upper chamber (3×10^5^/well) with serum-free medium and the lower chamber with medium containing 20% FCS. After 24 h, the cells migrating through the filter were dried for 10 min, fixed in absolute alcohol and stained with hematoxylin and eosin. Cells on the lower chamber were counted under a microscope at ×100. The experiment was repeated three times.

### Effects of ERK1/2 and PI3K/AKT Inhibitors on the Proliferation and Invasion of SK-BR-3 Cells Transfected with AdsiBMP9 Adenovirus

The SK-BR-3 cells were treated with 20 µM PD98059 (ERK1/2 inhibitor) or 20 µM LY294002 (PI3K/AKT inhibitor) for 30 min, and then with AdsiBMP9 or AdsiNC adenoviruses for indicated periods. The ERK1/2 and AKT expression was detected by western blot assay 30 min later, the cell invasion was detected 36 h later, and the cell proliferation was measured by MTT assay 72 h later.

### Animal Models

Female nude mice were randomly divided into three groups (n = 5 per group). SK-BR-3 cells treated with AdBMP9 or AdsiBMP9 for 36 h were collected and suspended in 150 µl of phosphate buffer solution (PBS) and separately inoculated subcutaneously into nude mice (2×10^7^cells per mouse). In the blank control group, 2×10^7^ untreated SK-BR-3 cells were inoculated subcutaneously.

Tumors were observable two weeks later. The tumor size was measured once every 5 days and the tumor volume (V; mm^3^) was then calculated as follow: π/6×(R_max_×R_min_)^ 2^, where R = tumor diameter. Mice were sacrificed 55 d later and the tumors were collected, fixed in buffered formaldehyde and cut into sections for further histomorphometrical and immunohistochemical assays.

### Immunohistochemistry (IHC)

IHC was performed as previously described (17). Paraffin-embedded tumors were cut into 4-µm sections which were then deparaffinized, rehydrated and heat-treated with citrate buffer as usual. Then, these sections were incubated with primary and secondary antibodies conjugated with the peroxidase sequentially. Visualization was done after incubation with 0.05% 3, 3-diaminobenzidine tetrachloride (DAB).

Anti-HER2 monoclonal antibody (human, 1:500), anti-phosphor-HER2 monoclonal antibody (human, 1:500), anti-phosphor-ERK1/2 monoclonal antibody (rabbit, 1:300), anti-phosphor-AKT monoclonal antibody (rabbit, 1:300) were used as the primary antibodies.

### Statistical Analysis

Data were expressed as means ± standard deviations (SD). All the data were analyzed with SPSS version 16.0 via one-way ANOVA and independent sample t-test. A value of P<0.05 was considered statistically significant.

## Results

### Expression of HER2 in SK-BR-3 Breast Cancer Cells and Preparation of Recombinant SK-BR-3/BMP9 and SK-BR-3/siBMP9 Cells

The HER2 expression in human SK-BR-3 breast cancer cells was detected by RT-PCR and western blot assay (triple negative MDA-MB-231 breast cancer cells as a control). The mRNA and protein HER2 expression was detectable in SK-BR-3 breast cells while absent in MDA-MB-231 cells (Figure 1A and B). These findings confirmed that SK-BR-3 breast cancer cells were HER2-positive.

**Figure 1:** Expression of HER2 in SK-BR-3 breast cancer cells and preparation of recombinant SK-BR-3/BMP9 and SK-BR-3/siBMP9 cells. (A) HER2 expression in SK-BR-3 cells and MDA-MB-231 cells was measured by RT-PCR and Western blot assay and preparation of recombinant SK-BR-3/BMP9 cells and SK-BR-3/siBMP9 cells. (B) SK-BR-3 cells transfected with different adenoviruses for 36 h under fluorescent microscope. (C) RT-PCR and (D) Western blot assay were performed to measure BMP9 expression in recombinant SK-BR-3/BMP9 cells and SK-BR-3/siBMP9 cells. All experiments were performed in triplicate. Bars represent SD. *P<0.05 vs. control group.

SK-BR-3 cells were transfected with BMP9-expressing adenoviruses (AdBMP9) and BMP9-siRNA adenoviruses (AdsiBMP9), respectively, to generate recombinant SK-BR-3/BMP9 and SK-BR-3/siBMP9 cells. The transfection efficiency of SK-BR-3 cells at 36 h was observed under fluorescence microscope (Figure 1C). RT-PCR and western blot assay showed that recombinant SK-BR-3/BMP9 and SK-BR-3/siBMP9 cells were well prepared for the subsequent experiments (Figure 1 D).

### BMP9 Inhibited the Proliferation and Metastasis of SK-BR-3 Cells in vitro

The viability of SK-BR-3 cells was analyzed by MTT assay and colony formation assay. MTT assay demonstrated that the proliferation of SK-BR-3/BMP9 cells was markedly inhibited in a time-dependent manner when compared with the SK-BR-3 cells and SK-BR-3/GFP cells (P<0.05), while the proliferation of SK-BR-3/siBMP9 cells significantly increased in a time-dependent manner (P<0.05) when compared with the SK-BR-3 cells and SK-BR-3/siNC cells (Figure 2A). Furthermore, colony formation assay showed that the colony-forming rate in SK-BR-3/BMP9 cells decreased by 34.8% (P<0.05) when compared with SK-BR-3 cells and SK-BR-3/GFP cells, and that in SK-BR-3/siBMP9 cells increased by 46.3% (P<0.05) when compared with SK-BR-3 cells and SK-BR-3/siNC cells (Figure 2B). These results suggest that BMP9 strongly suppresses the proliferation of SK-BR-3 cells.

**Figure 2:** BMP9 inhibited the proliferation, migration and invasiveness of SK-BR-3 cells. (A) MTT assay showed BMP9 suppressed the viability of SK-BR-3 cells. (B, C) Colony formation assay showed BMP9 inhibited the colony formation ability of SK-BR-3 cells (×100). (D, E) Wound-closure assay showed BMP9 inhibited the migration of SK-BR-3 cells (×100). (F, G) Transwell invasion assay showed that BMP9 inhibited the invasion of SK-BR-3 cells (×100). All experiments were performed in triplicate. Bars represent SD. *P<0.05 vs. control group.

Cell migration and invasion plays a crucial role in the tumor metastasis. Wound-closure and Transwell invasion assays were employed to detect the migration and invasion abilities mediated by BMP9. Results demonstrated the wound-closure rate of SK-BR-3/BMP9 cells decreased by 26.2% (P<0.05) and the invasive SK-BR-3/BMP9 cells decreased by 37.2% (P<0.05) when compared with SK-BR-3 cells and SK-BR-3/GFP cells. In addition, the wound-closure rate of SK-BR-3/siBMP9 cells increased by 28.1% and the invasive SK-BR-3/siBMP9 cells increased by 43.7% (P<0.05) when compared with SK-BR-3 cells and SK-BR-3/siNC cells (Figure 2C and D). These results suggest that BMP9 significantly suppresses the migration and metastasis abilities of SK-BR-3 cells.

### BMP9 Inhibited HER2 Activation and Down-regulated HER2 Expression through Inhibiting ERK1/2 (MAPK) and PI3K/AKT Pathways

Clinical studies have shown a strong relationship between HER2 expression and poor prognosis of breast cancer patients [2], [19]. Increased HER2 receptor expression is also associated with the aggressiveness and malignancy of breast cancer with high morbidity [2], [19]. Both total and phosphorylated HER2 proteins were detected by Western blot assay. Results indicated that BMP9 down-regulated the HER2 protein expression and inhibited the HER2 phosphorylation at the same time (Figure 3B). Furthermore, RT-PCR indicated that BMP9 inhibited the HER2 expression by suppressing the transcription of HER2 gene in SK-BR-3 cells (Figure 3A).

**Figure 3:** BMP9 inhibited HER2 activation and down-regulated HER2 expression through inhibiting the phosphorylation of MAPK and PI3K/AKT signaling pathways in SK-BR-3 breast cancer cells. (A) RT-PCR showed BMP9 inhibited HER2 mRNA expression in SK-BR-3 cells. (B) Western blot assay demonstrated BMP9 inhibited HER2 activation and decreased HER2 protein expression in SK-BR-3 cells. (C) Western blot assay demonstrated BMP9 inhibited ERK1/2 signaling in SK-BR-3 cells. (D) Western blot assay demonstrated BMP9 inhibited PI3K/AKT signaling in SK-BR-3 cells. All experiments were performed in triplicate. Bars represent SD. *P<0.05 vs. control group.

MAPK pathway is one of the major signaling pathways associated with cancer progression and metastasis [20], [21]. We investigated the effect of BMP9 on the MAPK signaling pathway. Western bolt assay demonstrated that BMP9 inhibited the phosphorylation of ERK1/2, but had no effect on the p38 and JNK expression in SK-BR-3 cells (Figure 3C). PI3K/AKT pathway is another major signaling pathway associated with cellular viability and invasion [22]–[24]. Western bolt assay demonstrated that BMP9 inhibited the phosphorylation of AKT in SK-BR-3 cells (Figure 3D).

### Effect of Inhibition of ERK1/2 and PI3K/AKT Signaling Pathways on the Proliferation and Metastasis of SK-BR-3 Cells Transfected with AdsiBMP9

We further confirmed the ERK1/2 and PI3K/AKT pathways were involved in the BMP9 mediated proliferation and metastasis of SK-BR-3 cells. Inhibitors of ERK1/2 (PD98059) or PI3K/AKT (LY294002) were used to pre-treat the SK-BR-3 cells for 30 min which were then transfected with AdsiBMP9 adenovirus. Results showed that AdsiBMP9 induced phosphorylation of ERK1/2 and AKT was reversed by PD98059 (P<0.05) and LY294002 (P<0.05) independently (Figure 4A and B). Then, the proliferation and metastasis were detected after addition of PD98059 or LY294002. Results showed that the proliferation and metastasis of SK-BR-3 cells after AdsiBMP9 transfection were reversed by PD98059 and LY294002 (Figure 4C and D). These results suggest that ERK1/2 and PI3K/AKT pathways are involved in the BMP9 mediated proliferation and metastasis of SK-BR-3 cells.

**Figure 4:** ERK1/2 and PI3K/AKT signaling pathways were involved in BMP9 mediated inhibition of proliferation and metastasis. (A) Effect of ERK1/2 inhibitor (PD98059) on the expression of ERK1/2 and phosphor-ERK1/2. (B) Effect of PI3K/AKT inhibitor (LY294002) on the expression of AKT and phosphor-AKT. SK-BR-3 cells were transfected with AdsiBMP9 in the present of PD98059 or LY294002 for 72 h (C) MTT assay showed that AdsiBMP9 induced proliferation was reversed by PD98059 and LY294002. (D) Transwell assay showed that the AdsiBMP9 induced invasion was reversed by PD98059 and LY294002. All experiments were performed in triplicate. Bars represent SD. *P<0.05 vs. control group.

### BMP9 Inhibited the Tumorigenesis of SK-BR-3 Cells in vivo

Our results suggested that BMP9 suppressed the proliferation and metastasis of SK-BR-3 cells *in vitro*. To confirm this effect *in vivo*, cells (SK-BR-3/siBMP9, SK-BR-3, SK-BR-3/BMP9) were subcutaneously inoculated into nude mice. The tumor was observed in SK-BR-3/siBMP9 group, SK-BR-3 group and SK-BR-3/BMP9 group on days 16, 19 and 23 after subcutaneously inoculation. Tumor volume was measured once every 5 days using a vernier caliper and the tumors were collected on day 55 (Figure 5A). The mean volume of tumors in SK-BR-3/siBMP9 group, SK-BR-3 group and SK-BR-3/BMP9 group was 1149±210 mm^3^, 268±136 mm^3^ and 65±12.8 mm^3^, respectively (Figure 5B). Histological examination (HE staining) showed that the tumor cells in three groups were all heterogeneous, the nuclei were enlarged, and the nucleus/cytoplasm ratio increased (Figure 5C). Immunohistochemistry (IHC) showed that there was a lower expression of HER2, p-HER2, p-ERK1/2 and p-AKT in SK-BR-3/BMP9 group when compared with SK-BR-3 group; while there was a higher expression of HER2, p-HER2, p-ERK1/2 and p-AKT in SK-BR-3/siBMP9 group, when compared with SK-BR-3 group (Figure 5D). These findings suggest that BMP9 suppresses the growth of SK-BR-3 cells and BMP9 inhibits the expression of HER2, ERK1/2, PI3K/AKT in SK-BR-3 cells *in vivo*.

**Figure 5:** Antitumor effect of BMP9 in breast cancer SK-BR-3 xenograft models. (A) On day 55, tumors were collected from three groups. (B) Tumor growth curve of three groups. Results showed BMP9 inhibited the growth of SK-BR-3 cells in vivo. (C) HE staining of the tumors in three groups (×400). (D) Immunohistochemistry of tumors in three groups (×400).

## Discussion

Human epidermal growth factor receptor 2 (HER2, also known as ErbB2) is expressed in approximately 30% of breast cancers and associated with increased mortality, shortened survival and relapse [3], [25], [26]. Elevated HER2 receptor plays a crucial role in promoting the cell growth, viability and invasion of HER2-positve breast cancer. Therefore, HER2 has been an important target for the breast cancer treatment. BMP9 has been shown to exert anti-tumorigenic effects in human prostate cancer, osteosarcoma and hepatocellular carcinoma [27], [28]. Our previous studies demonstrate that BMP9 inhibited the proliferation, migration and invasion of triple-negative MDA-MB-231 human breast cancer cells and promoted their apoptosis *in vitro* and *in vivo* [3]. In this study, our findings demonstrated that BMP9 has a dramatically inhibitory effect on the growth and metastasis of HER2-positive SK-BR-3 cells *in vitro* and *in vivo.*

Cell proliferation and invasiveness plays a crucial role in the tumorigenesis. Previous reports have shown that BMP9 as pleiotropic cytokine can significantly reduce the proliferation of MG-63 cells and HOS osteosarcoma cells in a time-dependent manner, and prevents the migration and invasiveness of prostate cancer [27]. In this study, we investigated the effect of BMP9 on the proliferation and metastasis in HER2-positvie SK-BR-3 breast cancer cells. Results showed that increased BMP9 expression inhibited the cell proliferation, colony formation, and migration, invasion of SK-BR-3 cells while silencing of BMP9 expression promoted the proliferation, colony formation, migration and invasion of SK-BR-3 cells. These findings suggested that BMP9 may function as a tumor suppressor in SK-BR-3 cells. However, the underlying mechanisms are still poorly understood.

Two major approaches for the treatment of HER2-positive cancers are to decrease the expression and activation of HER2 receptor [29], [30]. In this study, results showed that BMP9 down-regulated the HER2 protein expression and phosphorylation while both of them were significantly elevated in SK-BR-3 cells when BMP9 expression was silenced In addition, a significant down-regulation of HER2 mRNA expression was observed in BMP9 over-expression group while a dramatic up-regulation of HER2 mRNA expression in BMP9 silencing group. Based on above findings, we speculate that the inhibitory effect of BMP9 may be due to its inhibition on HER2 expression in SK-BR-3 cells. These findings suggest that BMP9 reduces the HER2 expression at mRNA and protein levels as well as inhibits the phosphorylation of HER2.

Phosphorylation of HER2 receptor tyrosine kinase activates the MAPK and PI3K/AKT signaling pathways, which in turn promotes the cell proliferation and metastasis [30]–[33]. MAPK and PI3K/AKT, which are major pathways involved in the malignant progression of various tumors, mediate the proliferation, migration and invasion of breast cancer. Our results showed that AdBMP9 transfection decreased the phosphorylation of ERK/12 whereas had no significant effect on the p38 and JNK. On the contrary, AdsiBMP9 transfection increased the phosphorylation of ERK1/2 while had no dramatic effect on the p38 and JNK. The findings also suggest that AdBMP9 decreases the phosphorylation of AKT while AdsiBMP9 increases the phosphorylation of AKT. These results demonstrate that BMP9 inhibits the activation of ERK1/2 and AKT.

To confirm that ERK1/2 and AKT pathways are involved in the BMP9 mediated inhibition of proliferation and metastasis of SK-BR-3 cells, cells were pre-treated with ERK/12 specific inhibitor (PD98059) or PI3K/AKT specific inhibitor (LY294002) for 30 min, and then transfected with AdsiBMP9 for 36 h. Results showed that the phosphorylation of ERK1/2 and AKT was inhibited by the specific inhibitors independently. AdsiBMP9 induced proliferation and invasion were reversed by these inhibitors, suggesting that BMP9 affects cell proliferation via the ERK1/2 and PI3K/AKT signaling pathways. These results are consistent with those from previous studies, demonstrating that ERK1/2 and PI3K/AKT signaling pathways play crucial roles in the proliferation and invasion of breast cancer cells [34], [35]. All these findings demonstrate that ERK1/2 and PI3K/AKT signaling pathways are involved in the BMP9 mediated inhibition of proliferation and invasion of SK-BR-3 cells.

Furthermore, the antitumor effect of BMP9 against SK-BR-3 breast cancer cells was also studied *in vivo*. Our results showed that AdBMP9 inhibited the tumor growth of SK-BR-3 xenografts *in vivo*, down-regulated the HER2 protein expression and inhibited the phosphorylation of HER2, ERK1/2, and AKT in the xenografts. On the other hand, opposite results were observed in AdsiBMP9 group. These results demonstrate that BMP9 inhibits the tumor growth and decreases the HER2 expression, and the phosphorylation of HER2, ERK1/2 and AKT in SK-BR-3 cells *in vivo*.

In conclusion, the BMP9 mediated inhibition of the proliferation and invasion of HER2-positive SK-BR-3 cells *in vitro* and *in vivo* are ascribed to the loss of HER2 activation and suppression of its downstream molecules, including the ERK1/2 and PI3K/AKT cascades. Therefore, BMP9 may be a novel agent for the treatment of HER2-positive breast cancers.

## References

[1] ZhangYJ (2012) The molecular subtype of breast cancer. Prac J Can 27: 98–100.

[2] SehdevV, LaiJC, BhushanA (2009) Biochanin A Modulates Cell Viability, Invasion, and Growth Promoting Signaling Pathways in HER-2-Positive Breast Cancer Cells. J Oncol 2009: 121458.2016909710.1155/2009/121458PMC2821773

[3] RossJS, SlodkowskaEA, SymmansWF, PusztaiL, RavdinPM, et al (2009) The HER-2 receptor and breast cancer: ten years of targeted anti-HER-2 therapy and personalized medicine. Oncologist 14: 320–368.1934629910.1634/theoncologist.2008-0230

[4] LaiHW, ChienSY, KuoSJ, TsengLM, LinHY, et al (2012) The Potential Utility of Curcumin in the Treatment of HER-2-Overexpressed Breast Cancer: An In Vitro and In Vivo Comparison Study with Herceptin. Evid Based Complement Alternat Med 2012: 486568.2187671310.1155/2012/486568PMC3162976

[5] MerkhoferEC, CogswellP, BaldwinAS (2010) Her2 activates NF-kappaB and induces invasion through the canonical pathway involving IKKalpha. Oncogene 29: 1238–1248.1994633210.1038/onc.2009.410PMC2829103

[6] FanP, McDanielRE, KimHR, ClagettD, HaddadB, et al (2012) Modulating therapeutic effects of the c-Src inhibitor via oestrogen receptor and human epidermal growth factor receptor 2 in breast cancer cell lines. Eur J Cancer 48: 3488–3498.2265832010.1016/j.ejca.2012.04.020PMC3518839

[7] GhoshR, NarasannaA, WangSE, LiuS, ChakrabartyA, et al (2011) Trastuzumab has preferential activity against breast cancers driven by HER2 homodimers. Cancer Res 71: 1871–1882.2132492510.1158/0008-5472.CAN-10-1872PMC3221734

[8] SlamonDJ, Leyland-JonesB, ShakS, FuchsH, PatonV, et al (2001) Use of chemotherapy plus a monoclonal antibody against HER2 for metastatic breast cancer that overexpresses HER2. N Engl J Med 344: 783–792.1124815310.1056/NEJM200103153441101

[9] Piccart-GebhartMJ, ProcterM, Leyland-JonesB, GoldhirschA, UntchM, et al (2005) Trastuzumab after adjuvant chemotherapy in HER2-positive breast cancer. N Engl J Med 353: 1659–1672.1623673710.1056/NEJMoa052306

[10] RomondEH, PerezEA, BryantJ, SumanVJ, GeyerCEJr, et al (2005) Trastuzumab plus adjuvant chemotherapy for operable HER2-positive breast cancer. N Engl J Med 353: 1673–1684.1623673810.1056/NEJMoa052122

[11] PegramMD, LiptonA, HayesDF, WeberBL, BaselgaJM, et al (1998) Phase II study of receptor-enhanced chemosensitivity using recombinant humanized anti-p185HER2/neu monoclonal antibody plus cisplatin in patients with HER2/neu-overexpressing metastatic breast cancer refractory to chemotherapy treatment. J Clin Oncol 16: 2659–2671.970471610.1200/JCO.1998.16.8.2659

[12] CobleighMA, VogelCL, TripathyD, RobertNJ, SchollS, et al (1999) Multinational study of the efficacy and safety of humanized anti-HER2 monoclonal antibody in women who have HER2-overexpressing metastatic breast cancer that has progressed after chemotherapy for metastatic disease. J Clin Oncol 17: 2639–2648.1056133710.1200/JCO.1999.17.9.2639

[13] WangK, FengH, RenW, SunX, LuoJ, et al (2011) BMP9 inhibits the proliferation and invasiveness of breast cancer cells MDA-MB-231. J Cancer Res Clin Oncol 137: 1687–1696.2189265210.1007/s00432-011-1047-4PMC11827914

[14] YeL, BokobzaSM, JiangWG (2009) Bone morphogenetic proteins in development and progression of breast cancer and therapeutic potential (review). Int J Mol Med 24: 591–597.1978719210.3892/ijmm_00000269

[15] LiB, YangY, JiangS, NiB, ChenK, et al (2012) Adenovirus-mediated overexpression of BMP-9 inhibits human osteosarcoma cell growth and migration through downregulation of the PI3K/AKT pathway. Int J Oncol 41: 1809–1819.2294823410.3892/ijo.2012.1617

[16] ReddiAH, ReddiA (2009) Bone morphogenetic proteins (BMPs): from morphogens to metabologens. Cytokine Growth Factor Rev 20: 341–342.1990083110.1016/j.cytogfr.2009.10.015

[17] WagnerDO, SieberC, BhushanR, BorgermannJH, GrafD, et al (2010) BMPs: from bone to body morphogenetic proteins. Sci Signal 3: mr1.2012454910.1126/scisignal.3107mr1

[18] MoasserMM (2007) The oncogene HER2: its signaling and transforming functions and its role in human cancer pathogenesis. Oncogene 26: 6469–6487.1747123810.1038/sj.onc.1210477PMC3021475

[19] RossJS, FletcherJA, LinetteGP, StecJ, ClarkE, et al (2003) The Her-2/neu gene and protein in breast cancer 2003: biomarker and target of therapy. Oncologist 8: 307–325.1289732810.1634/theoncologist.8-4-307

[20] KangMH, OhSC, LeeHJ, KangHN, KimJL, et al (2011) Metastatic function of BMP-2 in gastric cancer cells: the role of PI3K/AKT, MAPK, the NF-kappaB pathway, and MMP-9 expression. Exp Cell Res 317: 1746–1762.2157039210.1016/j.yexcr.2011.04.006

[21] AdeyinkaA, NuiY, CherletT, SnellL, WatsonPH, et al (2002) Activated mitogen-activated protein kinase expression during human breast tumorigenesis and breast cancer progression. Clin Cancer Res 8: 1747–1753.12060612

[22] MengQ, XiaC, FangJ, RojanasakulY, JiangBH (2006) Role of PI3K and AKT specific isoforms in ovarian cancer cell migration, invasion and proliferation through the p70S6K1 pathway. Cell Signal 18: 2262–2271.1683974510.1016/j.cellsig.2006.05.019

[23] ChaoX, ZaoJ, Xiao-YiG, Li-JunM, TaoS (2010) Blocking of PI3K/AKT induces apoptosis by its effect on NF-kappaB activity in gastric carcinoma cell line SGC7901. Biomed Pharmacother 64: 600–604.2094729010.1016/j.biopha.2010.08.008

[24] OsakiM, OshimuraM, ItoH (2004) PI3K-Akt pathway: its functions and alterations in human cancer. Apoptosis 9: 667–676.1550541010.1023/B:APPT.0000045801.15585.dd

[25] SeshadriR, FirgairaFA, HorsfallDJ, McCaulK, SetlurV, et al (1993) Clinical significance of HER-2/neu oncogene amplification in primary breast cancer. The South Australian Breast Cancer Study Group. J Clin Oncol 11: 1936–1942.810503510.1200/JCO.1993.11.10.1936

[26] SlamonDJ, ClarkGM, WongSG, LevinWJ, UllrichA, et al (1987) Human breast cancer: correlation of relapse and survival with amplification of the HER-2/neu oncogene. Science 235: 177–182.379810610.1126/science.3798106

[27] YeL, KynastonH, JiangWG (2008) Bone morphogenetic protein-9 induces apoptosis in prostate cancer cells, the role of prostate apoptosis response-4. Mol Cancer Res 6: 1594–1606.1892297510.1158/1541-7786.MCR-08-0171

[28] LiQ, GuX, WengH, GhafooryS, LiuY, et al (2013) Bone morphogenetic protein-9 induces epithelial to mesenchymal transition in hepatocellular carcinoma cells. Cancer Sci 104: 398–408.2328184910.1111/cas.12093PMC7657113

[29] ImaiK, TakaokaA (2006) Comparing antibody and small-molecule therapies for cancer. Nat Rev Cancer 6: 714–727.1692932510.1038/nrc1913

[30] KuoHP, HsuSC, OuCC, LiJW, TsengHH, et al (2013) Ganoderma tsugae Extract Inhibits Growth of HER2-Overexpressing Cancer Cells via Modulation of HER2/PI3K/Akt Signaling Pathway. Evid Based Complement Alternat Med 2013: 219472.2366211910.1155/2013/219472PMC3638576

[31] BaselgaJ, SwainSM (2009) Novel anticancer targets: revisiting ERBB2 and discovering ERBB3. Nat Rev Cancer 9: 463–475.1953610710.1038/nrc2656

[32] YangHL, LinKY, JuanYC, KumarKJ, WayTD, et al (2013) The anti-cancer activity of Antrodia camphorata against human ovarian carcinoma (SKOV-3) cells via modulation of HER-2/neu signaling pathway. J Ethnopharmacol 148: 254–265.2361902010.1016/j.jep.2013.04.023

[33] ZhouNN, TangJ, ChenWD, FengGK, XieBF, et al (2012) Houttuyninum, an active constituent of Chinese herbal medicine, inhibits phosphorylation of HER2/neu receptor tyrosine kinase and the tumor growth of HER2/neu-overexpressing cancer cells. Life Sci 90: 770–775.2252537210.1016/j.lfs.2012.03.035

[34] MengX, CaiC, WuJ, CaiS, YeC, et al (2013) TRPM7 mediates breast cancer cell migration and invasion through the MAPK pathway. Cancer Lett 333: 96–102.2335305510.1016/j.canlet.2013.01.031

[35] LinY, CuiH, XuH, YueL, XuH, et al (2012) Jolkinolide B induces apoptosis in MDA-MB-231 cells through inhibition of the PI3K/Akt signaling pathway. Oncol Rep 27: 1976–1980.2242655410.3892/or.2012.1717

